The article "A New Feature Analysis Approach to Selecting Channels of EEG for Fatigue Driving" was published in 2022. Journal: Comput Math Methods Med.

# A New Feature Analysis Approach to Selecting Channels of EEG for Fatigue Driving

**DOI:** 10.1155/2022/4640426

**Published:** 2022-10-04

**Authors:** Yiqi Liao, Pengpeng Shangguan, Yiran Peng, Taorong Qiu

**Affiliations:** School of Mathematics and Computer Sciences, Nanchang University, Nanchang, 330031 Jiangxi, China

## Abstract

Fatigued driving is a significant contributor to traffic accidents. There are some issues with common EEG data of 32 channels, 64 channels, and 128 channels, such as difficult acquisition, high data redundancy, and difficult practical application. A new channel selection method called ReliefF_SFS is proposed to address the problem of how to reduce the number of channels while maintaining classification accuracy. It combines the ReliefF algorithm and the sequential forward selection (SFS) algorithm. When only T6, O1, Oz, T4, P3, and FC3 are used, the classification accuracy under Theta_Std+FE combined with ReliefF_SFS achieves 99.45%. The strategy suggested in this paper not only ensures the recognition accuracy but also reduces the number of channels when compared to other models based on the same data set.

## 1. Introduction

Electroencephalogram (EEG) signals are spontaneous electrical activity of brain cells recorded by electrodes on the surface of the scalp, which are highly random. EEG signals record the electrical changes in brain activity and can directly reflect the fatigue state. There are two main categories of feature extraction methods based on EEG signals, including linear analysis methods and nonlinear analysis methods. Linear analysis methods mainly include time domain analysis methods, frequency domain analysis methods, and time-frequency domain analysis methods. Time domain analysis methods mainly include the extraction of features such as mean, median, variance, standard deviation, skewness, and kurtosis. The frequency domain analysis method mainly decomposes the EEG signal into multiple bands by wavelet transform or Fourier transform. Muhammad et al. [1] extracted the mean, variance, minimum, maximum, *δ*, *θ*, *α*, *β*, *γ*, and sample entropy of the ECG signal and used support vector machine(SVM) for classification. The accuracy of binary classification reached 80%. Nonlinear analysis methods mainly include the extraction of features such as entropy and fractal dimension. Ye et al. [2] proposed a fatigue driving state recognition method based on sample entropy and kernel principal component analysis, which combined the advantages of high recognition accuracy of sample entropy and strong processing capability of kernel principal component analysis in nonlinear principal component reduction and nonlinearity and achieved good results. Lin et al. [3] proposed a method for the dynamic construction of functional brain networks based on singular value entropy and fractal dimensionality. The experimental results showed that the method has high accuracy in fatigue driving recognition.

Although these methods perform better in feature extraction of EEG signals, most scholars only analyse EEG signals from a single aspect of linearity or nonlinearity, which is one-sided. Therefore, in this paper, the frequency domain features and fuzzy entropy features of the EEG signal are extracted separately, and the best performing subband features of the frequency domain features are fused with the fuzzy entropy features to form fused features, which are used as preparatory data for channel selection.

The 32-channel, 64-channel, and 128-channel EEG signal acquisition devices require electrodes to be arranged in various brain regions of the human brain, which is not only time-consuming and labour-intensive but also lacks relevance and convenience, as well as resulting in significant data redundancy and inefficient data processing. In the practical application of fatigue driving detection systems, due consideration should be given to the convenience and speed of EEG signal acquisition, the comfort of the driver, and the impact of the device on the driver's operation. Therefore, it is of practical importance to investigate the use of as few electrode channels as possible to detect the driver's driving status, not only to reduce the difficulty of EEG signal acquisition but also to improve the practicality.

Many scholars have conducted in-depth analysis and research on the channel selection of EEG signals in different fields. Zheng et al. [4] proposed a feature extraction and channel selection method of EEG signals for portable HCI systems for emotion recognition. This method was formed by extracting discriminative features of EEG signals in different dimensions and combining the relief algorithm, and the floating generalized sequential backward selection algorithm. The experimental results showed that the majority of the optimal channel set was located at the front end, and 10 channel EEG signals with extremely high accuracy were selected, with an average classification accuracy of 91.31% on both the self-collected and public datasets. Ru et al. [5] proposed a dynamic channel selection method based on channel location and EEG signal power spectral density and selected one of the channels with the strongest epilepsy detection ability as the feature extraction channel, so as to enhance the performance of epilepsy recognition and detection. Finally, 6 channels were selected from 21 channels, achieving a better performance of 98.99% accuracy, 98.52% sensitivity, and 99.52% specificity. Shoka et al. [6] proposed an automatic epilepsy diagnosis system based on EEG signal feature extraction and channel selection, which minimized the dimensionality by selecting the most affected channels through the variance parameter and finally reduced 23 channels to 3. Zhang et al. [7] proposed a ReliefF-Pearson based channel selection algorithm for olfactory EEG signals, combining the weighting idea of ReliefF and the correlation principle of Pearson. The results showed that the method was able to significantly reduce the number of channels while ensuring a certain classification accuracy. Praveena et al. [8] proposed a supervised classifier-based important feature selection method for seizure recognition, in which the ReliefF method was used to reduce the dimensionality of extracted features, and the long short-term memory (LSTM) method was used for classification. The results showed that the classification accuracy of the method was improved by 0.6%-16%.

In the field of fatigue driving, although there are researchers working on channel selection methods, they are still in the early stages of research, with few researchers or research results, and even more distant from practical applications. EEG signal channel selection for fatigue driving mainly includes single-channel selection and multichannel selection. Single-channel selection methods ensure a minimum number of channels, but ignore the fact that EEG signals from different drivers are different, resulting in poor detection results. The multichannel selection method ensures detection results with the lowest possible number of channels.

Hu [9] used a channel+feature+classifier approach applied to the fatigue driving dataset, and the selected combination of the CP4 channel, fuzzy entropy feature, and random forest classifier achieved 96.6% accuracy. Liu [10] proposed an adaptive multiscale sample entropy feature extraction algorithm based on empirical modal decomposition applied to the fatigue driving dataset and achieved 97.87% recognition accuracy on Fp1 and Fp2 electrodes. Chai et al. [11] used independent component analysis (ICA) and scalp map projection for EEG-based driver fatigue classification. The channels are reduced from 32 to 16, and the classification results of 16 channels are equivalent to those of 32 channels. Min et al. [12] proposed a feature extraction method of multi entropy fusion to select 10 channels of fatigue driving EEG data in 4 regions on an accuracy-based weight calculation method, which achieved 98.3% recognition accuracy.

The above studies show channel selection has practical significance in the field of fatigue driving. However, how to reduce the number of EEG signal channels as much as possible while improving the recognition accuracy still requires continuous research. Therefore, this paper focuses on the study of multichannel selection methods. Based on the extracted different EEG signal feature data, combined with the weight calculation of ReliefF algorithm and the feature selection of SFS algorithm, a channel selection method based on ReliefF_SFS is proposed to explore the use of as few EEG signal channels as possible to achieve a high recognition accuracy. It not only reduces redundant channels but also improves the practicality of fatigue detection in the driving field.

The rest of the paper is organized as follows: Section 2 introduces the relevant theory and methods of the proposed method.  Section 3 focuses on the feature extraction part of channel selection.  Section 4 introduces the channel selection algorithm with ReliefF_SFS on different features.  Section 5 presents the experiments and analyses the results.  Section 6 summarizes the paper.

## 2. Relevant Theory and Methods

### 2.1. Frequency Domain Features

A large amount of EEG signal feature information is reflected in the frequency features, and extracting the frequency domain features after wavelet decomposition of EEG signals is a common analysis method. Wavelet packet decomposition (WPD) [13] is a mainstream signal analysis method that has been widely used in various signal-related fields, including medical diagnosis, metal detection, and natural disaster signal analysis. WPD can decompose and reconstruct a signal into multiple signal components with the same bandwidth but different center frequencies. WPD can provide higher accuracy in the high frequency part of the signal and no redundant or missing information. WPD has a strong ability to decompose nonstationary signals to obtain multiscale signals. Therefore, it is commonly used for signal feature extraction. Equation (1) is used for wavelet packet decomposition of EEG signal.

(1) $$\begin{array}{c} \left\{\begin{array}{c} w_{\left(2n\right)}\left(x\right)=\sqrt{2}\underset{k\in Z}{\sum }h_{k}w_{n}\left(2x-k\right),\\ w_{\left(2n+1\right)}\left(x\right)=\sqrt{2}\underset{k\in Z}{\sum }g_{k}w_{n}\left(2x-k\right), \end{array}\right. \end{array}$$

where *h*_*k*_ is a low-pass filter bank and *g*_*k*_ is a high-pass filter bank. The wavelet packet decomposition is a collection of functions with certain connections, including scale functions *W*_0_(*x*) = *Φ*(*x*) and wavelet functions *W*_1_(*x*) = *φ*(*x*).The WPD method can decompose both low frequency signals and high frequency signals at the same time and is more efficient than the wavelet transform [14] for feature extraction.

In the experiments of this paper, firstly, the sampling frequency of EEG signal was reduced to 128 Hz, secondly, a six-layer wavelet packet decomposition tree was built, and then the original EEG signal was decomposed into four subbands, including Theta subband (4-8 Hz), Alpha subband (8-13 Hz), Beta1 subband (13-20 Hz), and Beta2 subband (20-30 Hz). Finally, the standard deviation (Std) features are extracted for each subband, and the best performing subband features are fused with the fuzzy entropy features to form the fused features. The standard deviation is a measure of the dispersion of the data and is calculated as

(2) $$\begin{array}{c} F=\sqrt{\frac{1}{N_{s}}\overset{N_{s}}{\underset{i=1}{\sum }}{\left(x\left(i\right)-\overset{¯}{x}\right)}^{2}}, \end{array}$$

where *x*(*i*) denotes the time series and *N*_*s*_ denotes the size of the time series.

### 2.2. FE

The concept of fuzzy entropy (FE) was first proposed by Chen et al. [15] in 2007. FE describes the fuzziness of a fuzzy set [16] and measures the probability of a new pattern being generated. The larger the measure, the greater the probability of the new pattern being generated and the greater the sequence complexity. The specific algorithm is described as follows:

**Step 1 .**

Given a time series.

(3) $$\begin{array}{c} \left\{X\left(i\right),i=1,2,\cdots ,n\right\}. \end{array}$$

**Step 2 .**

Dividing the time series into *k* = *n* − *m* + 1 series with a window of *m*.

(4) $$\begin{array}{c} X_{i}\left(t\right)=\left(x_{i}\left(t\right),x_{i+1}\left(t\right),\cdots ,x_{i+m-1}\left(t\right)\right). \end{array}$$

**Step 3 .**

Calculate the distance between each sequence and all *k* sequences.

(5) $$\begin{array}{c} d_{ij}=\max\left|x_{i+k}\left(t\right)-x_{j+k}\left(t\right)\right|,k=0,1,\cdots ,m-1. \end{array}$$

Matrix obtained.

(6) $$\begin{array}{c} \begin{array}{c} 1\\ 2\\ \cdots \\ \text{j}\\ \cdots \\ k \end{array}\begin{array}{c} 1\;2\;\cdots \;i\;\cdots \;k\\ \left[\begin{array}{cccccc} d_{1,1} & d_{2,1} & \cdots & \cdots & \cdots & \cdots \\ d_{1,2} & d_{2,2} & \cdots & \cdots & \cdots & \cdots \\ \cdots & \cdots & \cdots & \cdots & \cdots & \cdots \\ \cdots & \cdots & \cdots & d_{i,j} & \cdots & \cdots \\ \cdots & \cdots & \cdots & \cdots & \cdots & \cdots \\ \cdots & \cdots & \cdots & \cdots & \cdots & d_{k,k} \end{array}\right] \end{array}. \end{array}$$

**Step 4 .**

Calculation of fuzzy affiliation based on distance *d*.

(7) $$\begin{array}{c} D_{ij}^{m}=\mu \left(d_{ij}^{m},n,r\right)=\exp\left(\frac{-{\left(d_{ij}^{m}\right)}^{n}}{r}\right). \end{array}$$

Averaging over all affiliations except itself.

(8) $$\begin{array}{c} \phi^{m}\left(n,r\right)=\frac{1}{N-m}\overset{N-m}{\underset{j=i}{\sum }}\left(\frac{1}{N-m-1}\overset{N-m}{\underset{j=1,j\neq i}{\sum }}D_{ij}^{m}\right). \end{array}$$

**Step 5 .**

Grow the window *m* to *m* + 1 and repeat steps 2 to 4.

**Step 6 .**

Calculation of fuzzy entropy.

(9) $$\begin{array}{c} \text{FuzzyEn}\left(t\right)=\text{In}\Phi^{m}\left(t\right)-\text{In}\Phi^{m+1}\left(t\right). \end{array}$$

In this paper, the fuzzy entropy is calculated by taking *m* as 2 and *r* as 0.25.

### 2.3. ReliefF

The Relief algorithm was first proposed by Kira and Rendell [17] in 1992. Relief is a feature weighting algorithm that assigns different weights to features based on the correlation between features and categories. The correlation between features and categories in the Relief algorithm is based on the ability of features to discriminate close samples. The Relief algorithm is simple and efficiently, which has been widely used. However, it has some limitations as it can only handle two categories of data. Therefore, Kononenko [18] extended it to obtain the ReliefF algorithm in 1994, which can handle multicategory problems. This algorithm is used to deal with regression problems where the target attributes are continuous values. The larger the feature weights, the better its classification performance. The ReliefF algorithm [8] is described in Algorithm 1.

In this paper, the weights are calculated as 80 for *m*, 10 for *k*, and 30 for *N*.

### 2.4. SFS

The sequential forward selection (SFS) algorithm [19] is used to reduce the initial d-dimensional feature space to a k-dimensional feature subspace, where <*d* . The algorithm can be described as follows: the feature subset *X* starts from the empty set and one feature *x* at a time is selected to be added to the feature subset *X* such that the feature function *Y*(*X*) is optimal. In simple terms, this means that one feature is chosen at a time that makes the evaluation function optimal and is a simple greedy algorithm.

In this paper, the characteristic function is defined as

(10) $$\begin{array}{c} Y\left(X\right)=\text{Acc}=\frac{\text{TP}+\text{TN}}{\text{TP}+\text{TN}+\text{FP}+\text{FN}} \end{array}$$

where Acc indicates accuracy, TP indicates positive samples predicted by the model as positive class, TN indicates negative samples predicted by the model as negative class, FP indicates negative samples predicted by the model as positive class, and FN indicates positive samples predicted by the model as negative class.

The SFS algorithm is described in Algorithm 2.

### 2.5. KNN

The K-Nearest Neighbor (KNN) classification algorithm was originally proposed by Silverman et al. [20] in 1951 and later modified by Cover and Hart [21] in 1967. The KNN classifier is a simple and general classification method. Due to its simplicity and robustness, it has been widely used in a number of fields, including pattern recognition, model ranking, and text classification. KNN is a nonparametric lazy learning algorithm, whose algorithm principle is that when a new value *X* is predicted, the class of *X* is determined based on the class of the *K* nearest points to it.

The two most important processes in this algorithm are the calculation of point distances and the selection of *K* values. In the distance calculation process, the KNN algorithm uses the Euclidean distance, which is calculated in two dimensions as.

(11) $$\begin{array}{c} \rho =\sqrt{{\left(x_{2}-x_{1}\right)}^{2}+{\left(y_{2}-y_{1}\right)}^{2}}. \end{array}$$

In the process of selecting the *K* value, the cross-validation starts from selecting a smaller *K* value and keeps increasing the value of *K*. The variance of the validation set is then calculated, and a more appropriate value of *K* is finally found [22].

In this paper, *K* was taken to be 10.

## 3. Feature Extraction

### 3.1. Data Collection

The experimental data were collected mainly through a vehicle driving simulator (ZY-31D Vehicle Driving Simulator, Beijing Zhongyulai Fit Teaching Equipment Co., Ltd.) and a set of 32-channels EEG signal electrode caps (sampling frequency 1000 Hz). The position of the 32 electrodes in the electrode cap according to the 10-20 international standard is shown in Figure 1.

In the experimental data collection process, firstly, subjects were simulated to drive for 20 minutes using a vehicle driving simulator, and the last 5 minutes of data were recorded as resting state data (recorded as JX), then, subjects drove continuously for more than 1 hour, and the Fatigue Scale-14 (FS-14) [23] was used to determine the driver's state until the subject's brain was in a fatigued state, and the last 5 minutes of data were recorded as fatigue state data (recorded as ZD). The final EEG data were collected for 300 seconds each in the resting and fatigued states, with a sampling frequency of 1000 Hz and 32 channels. In the actual processing, the two reference electrode data (A1 and A2) were removed. The final experimental data was obtained for 600 seconds and 30 channels for each subject.

The names of the electrodes correspond to their positions as follows: Fp1 (1), Fp2 (2), F7 (3), F3 (4), Fz (5), F4 (6), F8 (7), FT7 (8), FC3 (9), FCz (10), FC4 (11), FT8 (12), T3 (13), C3 (14), Cz (15), C4 (16), T4 (17), TP7 (18), CP3 (19), CPz (20), CP4 (21), TP8 (22), T5 (23), P3 (24), Pz (25), P4 (26), T6 (27), O1 (28), Oz (29), and O2 (30).

Firstly, after acquiring the resting-state data and fatigue state data, we divided each part of the resting-state data or fatigue state data into 1 second and formed them together. Then, we splice the processed resting-state data and fatigue-state data into a complete dataset. During the training and testing period, the whole dataset is shuffled and divided into the training set and the testing set.

### 3.2. Feature Matrix Construction

In this paper, experimental data from 10 people were collected at a sampling frequency of 1000 Hz for 300 seconds each in the resting and fatigue states to construct the experimental samples, using 10-20 international standards for 30 channels (removing the two reference electrodes). For each individual, this constitutes a sample matrix of (2 × 300 × 1000) × 30 and for 10 individuals, a sample matrix of (2 × 10 × 300 × 1000) × 30, where (2 × 10 × 300 × 1000) represents the size of the rows of the sample matrix and 30 represents the number of channels. The total sample size is 6,000,000 (including 3,000,000 resting state samples and 3,000,000 fatigue state samples), and the number of channels is 30.

#### 3.2.1. Construction of a Single Feature Matrix

Based on the selected experimental samples, the feature extraction is divided into 1000 data per second in the extraction process of frequency domain features and fuzzy entropy features.

For each feature, each subject gets a 300 × 30 resting state feature sample matrix *X*_*JX*_ and a 300 × 30 fatigue state feature sample matrix *X*_*ZD*_, as shown in Equations (12) and (13), where *x*_*i*,*j*_ denoting the feature value. 10 subjects get a (10 × 300) × 30 resting state feature sample matrix and a (10 × 300) × 30 fatigue state feature sample matrix, where 10 × 300 represents the size of the matrix rows and 30 represents the number of channels, that is 3000 resting state samples and 3000 fatigue state samples were obtained after feature extraction, and the number of channels was 30, as preparatory data for subsequent channel selection.

(12) $$\begin{array}{c} \begin{array}{c} 1\\ 2\\ \cdots \\ 300 \end{array}\begin{array}{c} \begin{array}{cccc} 1 & 2 & \cdots & 30 \end{array}\\ \left[\begin{array}{cccc} x_{1,1} & x_{1,2} & \cdots & x_{1,30}\\ x_{2,1} & x_{2,2} & \cdots & x_{2,30}\\ \cdots & \cdots & \cdots & \cdots \\ x_{300,1} & x_{300,2} & \cdots & x_{300,30} \end{array}\right] \end{array}=X_{JX}, \end{array}$$

(13) $$\begin{array}{c} \begin{array}{c} 1\\ 2\\ \cdots \\ 300 \end{array}\begin{array}{c} \begin{array}{cccc} 1 & 2 & \cdots & 30 \end{array}\\ \left[\begin{array}{cccc} x_{1,1} & x_{1,2} & \cdots & x_{1,30}\\ x_{2,1} & x_{2,2} & \cdots & x_{2,30}\\ \cdots & \cdots & \cdots & \cdots \\ x_{300,1} & x_{300,2} & \cdots & x_{300,30} \end{array}\right] \end{array}=X_{ZD}. \end{array}$$

#### 3.2.2. Construction of the Fusion Feature Matrix

Firstly, the best performing frequency domain features are extracted from the different decomposed bands. For descriptive purposes, the Std feature extracted from the Theta subband is recorded as Theta_Std. Secondly, fuse the best performing frequency domain features with the FE features (e.g., Theta_Std+FE feature).

The resting-state fusion feature matrix *Y*_*JX*_ and the fatigue-state fusion feature matrix *Y*_*ZD*_ obtained when two single features are fused are shown in Equations (14) and (15), respectively, where *x*_*i*,*j*_ and *y*_*i*,*j*_ denote the feature value of the different features, respectively.

(14) $$\begin{array}{c} \begin{array}{c} 1\\ 2\\ \cdots \\ 300 \end{array}\begin{array}{c} \begin{array}{cccc} 1 & 2 & \cdots & 30 \end{array}\\ \left[\begin{array}{ccccccc} x_{1,1} & y_{1,1} & x_{1,2} & y_{1,2} & \cdots & x_{1,30} & y_{1,30}\\ x_{2,1} & y_{2,1} & x_{2,2} & y_{2,2} & \cdots & x_{2,30} & y_{2,30}\\ \cdots & \cdots & \cdots & \cdots & \cdots & \cdots & \cdots \\ x_{300,1} & y_{300,1} & x_{300,2} & y_{300,2} & \cdots & x_{300,30} & y_{300,30} \end{array}\right] \end{array}=Y_{JX}, \end{array}$$

(15) $$\begin{array}{c} \begin{array}{c} 1\\ 2\\ \cdots \\ 300 \end{array}\begin{array}{c} \begin{array}{cccc} 1 & 2 & \cdots & 30 \end{array}\\ \left[\begin{array}{ccccccc} x_{1,1} & y_{1,1} & x_{1,2} & y_{1,2} & \cdots & x_{1,30} & y_{1,30}\\ x_{2,1} & y_{2,1} & x_{2,2} & y_{2,2} & \cdots & x_{2,30} & y_{2,30}\\ \cdots & \cdots & \cdots & \cdots & \cdots & \cdots & \cdots \\ x_{300,1} & y_{300,1} & x_{300,2} & y_{300,2} & \cdots & x_{300,30} & y_{300,30} \end{array}\right] \end{array}=Y_{ZD}. \end{array}$$

## 4. Channel Selection Model Construction and Algorithm Description

### 4.1. Channel Selection Model Construction Based on ReliefF_SFS

The ReliefF method is a widely used feature selection method in classification problems, which has the advantages of simple computation and high operational efficiency. However, the ReliefF method only gets the weight of the feature, which can only evaluate the contribution value of the feature to the classification and cannot help delete the redundant feature [24]. The SFS method determines the optimal feature subset by selecting one feature at a time that results in the optimal value of the evaluation function. Therefore, this paper proposes a channel selection method based on ReliefF and SFS methods (recorded as ReliefF_SFS method) by combining the weight calculation properties of ReliefF method and the feature selection properties of SFS method. The method firstly uses the ReliefF method to calculate the channel weights of the EEG signals after feature extraction, secondly uses the SFS method to iteratively select the channel with the largest weight to join the channel subset (the channel subset starts from the empty set), and then uses a KNN classifier to perform five-fold cross-validation for each channel subset to obtain the recognition accuracy (i.e., the value of the feature function) for each channel subset. Finally, the optimal number of channels is determined based on the recognition accuracy. This method not only solves the problem of redundancy of EEG signal channels but also reduces the data dimensionality and facilitates the acquisition of signals and data processing.  Figure 2 shows the model construction process of the method.

Figure 2 includes the following main sections:

1. *EEG Signal Data Acquisition*. The EEG signal data set is obtained by acquisition with specialised equipment. (The specific method is shown in Section 3.1)
2. *EEG Signal Feature Extraction*. The frequency domain features, fuzzy entropy features, and fusion features of all channels were extracted for each S-second data of *R* subjects in the EEG signal data set in resting and fatigue states, respectively, as shown in Section 3.2. The obtained feature data were used as the preparatory data for channel selection
3. *Weighting Calculation*. Based on the extracted full-channel EEG signal feature data, the ReliefF method was used for channel weight calculation
4. *Channel Subset Selection*. Using the SFS method, the channel subset starts from the empty set, and the channel data with the largest weight is selected to join the channel subset each time. The channel subset is constructed iteratively
5. *Recognition Test*. For each channel subset, five-fold cross-validation was used to randomly select 80% of the data as the training set and the remaining 20% as the test set. The recognition accuracy of each channel subset was calculated separately based on the KNN classifier, and the optimal channel subset was determined by the recognition accuracy. The recognition accuracy and channel selection results of different features were compared to obtain the optimal combination of features+accuracy+channels number

### 4.2. Channel Selection Algorithm Based on a Single Feature Combined with ReliefF_SFS

In this section we focus on the channel selection algorithm based on single feature combined with ReliefF_SFS. The single features described here are the Std features of the Theta, Alpha, Beta1, and Beta2 subbands (recorded as Theta_Std, Alpha_Std, Beta1_Std, and Beta2_Std, respectively) and the FE feature. The algorithm is described in detail as shown in Algorithm 3.

### 4.3. Channel Selection Algorithm Based on Fusion Features Combined with ReliefF_SFS

In this section, the best performing subband features selected from the frequency domain features in Section 4.2 are fused with FE features before ReliefF_SFS channel selection, and the fusion method is shown in Section 3.2.2.

The overall process is similar to the channel selection algorithm based on a single feature in Section 4.2. However, different from being based on a single feature, the fusion features requires the construction of the fusion feature matrix.

For the selected optimal frequency domain features and fuzzy entropy features are fused to obtain the fusion feature matrix *F*1_(2 × *R* × *S*)×*x*×*N*_, where 2 × *R* × *S* represents the size of the matrix *F*1 rows, i.e. the number of samples, *N* represents the number of electrodes, i.e. the number of channels, and *x* represents the fusion feature amount (*x* = 2), i.e. the number of features extracted from each channel.

After obtaining the fusion feature matrix, the ReliefF_SFS is used for channel subset selection.

## 5. Experiments and Analysis of Results

### 5.1. Validity Test Based on a Single Feature Combined with ReliefF_SFS

*(1) Validity Test Based on Frequency Domain Features Combined with ReliefF_SFS*.  Table 1 shows the results of the four frequency domain feature data (Theta_Std, Alpha_Std, Beta1_Std, and Beta2_Std) sorted by channel weight value from largest to smallest.  Table 2 shows the recognition accuracy of each channel subset obtained from the four frequency domain feature data based on the ReliefF_SFS method after classification and recognition using a KNN classifier.  Figure 3 shows the optimal recognition accuracy and the corresponding number of channels obtained from the four frequency domain feature data after being processed by the ReliefF_SFS channel selection method.

As can be seen from Table 2 and Figure 3, the channel selection method based on Theta_Std features combined with ReliefF_SFS achieves a maximum recognition accuracy of 99.42% when using the 15 channels with the highest weights; the channel selection method based on Alpha_Std features combined with ReliefF_SFS achieves a maximum recognition accuracy of 91.73% when using the 19 channels with the highest weights; the channel selection method based on Beta1_Std features combined with ReliefF_SFS achieved a maximum recognition accuracy of 97.00% when using the 17 channels with the highest weights; the channel selection method based on Beta2_Std features combined with ReliefF_SFS achieved a maximum recognition accuracy of 86.70% when using the 20 channels with the highest weights. The experimental results show that the channel selection method based on Theta_Std features combined with ReliefF_SFS achieves up to 99.42% classification accuracy when using the 15 channels with the highest weights named (numbered) as T6 (27), O1 (28), Oz (29), T4 (17), P3 (24), FC3 (9), F7 (3), Fp2 (2), F3 (4), TP7 (18), TP8 (22), Cz (15), FT7 (8), Fz (5), and CP3 (19). And for each feature data when combined with the ReliefF_SFS method for channel selection, a subset of channels with *n* < 30 can be selected so that the feature function *Y*(*n*) reaches the maximum.

*(2) Validity Testing Based on Fuzzy Entropy Features Combined with ReliefF_SFS*.  Table 3 shows the results obtained by sorting the FE feature data according to the channel weight values from largest to smallest.  Table 4 shows the recognition accuracy of each channel subset obtained from the FE feature data based on the ReliefF_SFS method after classification and recognition using a KNN classifier. From Table 4, it can be seen that the channel selection method based on FE features combined with ReliefF_SFS achieves 99.22% classification accuracy when using the 7 channels with the highest weights named (numbered) as O1 (28), T6 (27), FC3 (9), Oz (29), TP8 (22), T4 (17), and P3 (24).

### 5.2. Validity Testing Based on Fusion Features Combined with ReliefF_SFS

Table 5 shows the results obtained by sorting the fused feature data Theta_Std+FE according to the average channel weight value from largest to smallest.  Table 6 shows the recognition accuracy of each channel subset obtained from the fused feature data Theta_Std+FE based on the ReliefF_SFS method after classification and recognition using a KNN classifier. From Table 6, it can be seen that the channel selection method based on Theta_Std+FE features combined with ReliefF_SFS achieves 99.45% classification accuracy when using the 6 channels with the highest weights named (numbered) as T6 (27), O1 (28), Oz (29), T4 (17), P3 (24), and FC3 (9).

### 5.3. Comparative Analysis

The EEG data were extracted in the frequency domain, fuzzy entropy, and fusion features, and then processed using the ReliefF_SFS channel selection method proposed in this paper, and the accuracy and number of channels obtained are shown in Table 7. As can be seen from Table 7, the channel selection method based on Theta_Std+FE features combined with ReliefF_SFS has the best performance in terms of both the number of channels and accuracy, with 99.45% classification accuracy when only six channels (T6, O1, Oz, T4, P3, and FC3) are used.

At the same time, by using the algorithm in this paper and the algorithm in other papers for fatigue driving status recognition experiments under the same data set, it is concluded that the proposed method in this paper has reduced the number of channels and improved the accuracy, which proves that the proposed method in this paper is feasible. This is because there may be redundant or unimportant data in the full channel data, resulting in a lower accuracy rate when using the full channel data for driver fatigue recognition.  Table 8 lists some of the compared methods and their corresponding channel numbers and recognition accuracies. It can be seen that the proposed channel selection method based on Theta_Std+FE features combined with ReliefF_SFS has the best recognition accuracy.

### 5.4. Subject-Specific Validity of Selected Channels

To verify the subject-specific validity of channel selection with Relief_SFS, we draw the brain topographic maps for the selected subjects. The specific process is as follows:

Firstly, we first randomly select 5 subjects from the dataset; secondly, for each subject, we calculate the specific features (which include frequency domain features, fuzzy entropy features, and fusion features) for each channel. Thirdly, we normalize the selected features and then draw their brain topographic map.

Figure 4 shows the brain topographic map of each subject based on the frequency domain features.  Figure 5 shows the brain topographic map of each subject based on the fuzzy entropy features.  Figure 6 shows the brain topographic map of each subject based on the fusion features.

Each row in the figure represents the performance of the resting and fatigue states of each subject selected for the different normalized features of the brain topography. Among them, JX1 and ZD1 represent the brain topography of the first subject's resting and fatigue state under each channel, respectively. Other symbols are in the same way. The darker the area of the graph, the greater the feature value of the channel.

As can be seen from Figures 4–6, overall, the channel area with the highest weights based on different features varies among states. The variation in features of the selected channels by our method is more obvious for different features. This also validates that the channels chosen by our approach are significant.

## 6. Conclusion

In this paper, a channel selection model based on ReliefF_SFS is proposed by extracting different features of EEG signals and combining the weight calculation of the ReliefF algorithm and the feature selection of the SFS algorithm. The experimental results show that the channel selection method proposed in this paper is feasible, and the number of channels is reduced while the recognition accuracy is guaranteed, which is of great significance for the implementation of practical applications.

## Figures and Tables

**Figure 1:** Electrode distribution.

**Figure 2:** Construction of channel selection model based on ReliefF_SFS method.

**Figure 3:** Optimal recognition accuracy and corresponding number of channels for four types of frequency domain feature data.

**Figure 4:** Brain topographic map of each subject based on the frequency domain features.

**Figure 5:** Brain topographic map of each subject based on the fuzzy entropy features.

**Figure 6:** Brain topographic map of each subject based on the combined features.

**Algorithm 1:** ReliefF.

**Algorithm 2:** SFS.

**Algorithm 3:** Channel selection algorithm based on a single feature combined with ReliefF_SFS.

**Table 1:** Sorting table of channel weights for frequency domain feature data (1 × 10^−3.^).

Theta_Std		Alpha_Std		Beta1_Std		Beta2_Std	
Number	Weight	Number	Weight	Number	Weight	Number	Weight
27	197.0	13	11.62	27	11.62	28	5.663
28	181.9	28	11.22	28	11.22	29	4.153
29	157.4	17	11.05	29	11.05	30	3.667
17	122.7	1	10.62	17	10.62	13	3.023
24	117.7	30	8.951	3	8.951	17	2.995
9	110.5	8	8.742	22	8.742	23	2.678
3	103.7	29	7.583	9	7.583	3	2.627
2	102.8	3	7.008	13	7.008	27	2.622
4	100.4	22	6.310	24	6.310	1	2.521
18	100.1	2	5.644	1	5.644	18	2.506
22	97.61	12	5.529	2	5.529	12	2.434
15	96.24	23	4.691	30	4.691	22	2.347
8	95.16	18	4.493	18	4.493	8	2.214
5	91.46	9	4.156	5	4.156	9	2.073
19	88.32	7	4.009	19	4.009	2	1.817
10	84.71	27	3.829	8	3.829	11	1.738
23	83.43	4	3.587	11	3.587	7	1.682
11	83.02	26	3.270	15	3.270	24	1.533
6	82.45	24	3.189	10	3.189	19	1.490
30	81.99	11	3.154	6	3.154	4	1.420
7	81.39	16	2.348	23	2.348	26	1.362
13	77.23	14	2.252	7	2.252	25	1.294
16	75.23	19	2.153	4	2.153	14	1.160
1	74.43	25	2.151	12	2.151	6	1.155
21	67.56	5	2.128	14	2.128	16	1.088
14	63.10	6	2.044	16	2.044	20	1.076
20	60.28	15	1.998	21	1.998	15	1.021
26	59.70	21	1.855	26	1.855	5	0.988
12	59.26	20	1.643	25	1.643	21	0.940
25	56.50	10	1.627	20	1.627	10	0.744

**Table 2:** Recognition accuracy of each channel subset based on KNN classifier (Unit: %).

Number of channels	Theta_Std	Alpha_Std	Beta1_Std	Beta2_Std
1	77.22	54.90	68.53	58.60
2	90.37	67.92	82.90	69.37
3	94.73	78.67	90.88	72.92
4	96.35	84.23	93.03	78.33
5	96.63	86.38	94.07	79.92
6	99.37	87.85	94.63	82.65
7	99.35	88.60	95.95	82.60
8	99.28	89.77	95.78	83.65
9	99.33	89.98	96.25	84.32
10	99.33	89.85	96.30	84.80
11	99.28	90.72	96.43	85.45
12	99.37	90.90	96.60	85.87
13	99.30	91.07	96.82	85.20
14	99.32	91.02	96.83	86.53
15	99.42	91.10	96.72	85.72
16	99.35	91.45	96.63	85.92
17	99.35	91.28	97.00	86.13
18	99.33	91.12	96.73	85.55
19	99.22	91.73	96.92	85.92
20	99.33	91.57	96.78	86.70
21	99.30	91.57	96.88	85.92
22	99.27	91.37	96.88	86.08
23	99.27	91.70	96.80	85.97
24	99.20	91.40	96.80	86.10
25	99.22	91.52	96.90	85.92
26	99.22	91.55	96.97	85.87
27	99.23	91.57	96.83	85.92
28	99.22	91.27	96.83	85.73
29	99.25	91.65	96.82	85.87
30	99.23	91.38	96.98	85.97

**Table 3:** Sorting table of channel weights for FE feature data (1 × 10^−4^).

Number	28	27	9	29	22	17	24	18	6	1
Weight	138	129.6	103.2	101	92.37	91.76	86.97	84.73	80.34	78.70
Number	10	16	19	4	13	23	15	3	5	11
Weight	78.06	75.13	73.57	73.05	72.22	71.33	67.84	67.72	67.55	66.70
Number	12	2	30	8	21	14	7	20	26	25
Weight	65.72	65.40	64.63	63.30	60.89	59.08	58.66	50.66	50.00	48.60

**Table 4:** Recognition accuracy of each channel subset based on KNN classifier (Unit: %).

Number of channels	1	2	3	4	5	6	7	8	9	10
FE	70.83	92.25	97.17	98.78	98.88	99.10	99.22	99.13	99.12	99.22
Number of channels	11	12	13	14	15	16	17	18	19	20
FE	99.13	99.15	98.92	99.08	99.10	99.07	99.10	99.05	99.07	99.03
Number of channels	21	22	23	24	25	26	27	28	29	30
FE	99.07	99.07	99.07	99.12	99.22	99.08	99.07	99.00	99.08	99.05

**Table 5:** Sorting table of average channel weights for Theta_Std+FE fusion feature data (1 × 10^−3^).

Number	27	28	29	17	24	9	3	2	18	4
Weight	105	97.85	83.77	65.94	63.21	60.42	55.24	54.66	54.28	53.86
Number	22	15	8	5	19	10	23	6	11	30
Weight	53.42	51.51	50.74	49.11	47.84	46.26	45.28	45.24	44.85	44.23
Number	7	13	16	1	21	14	12	20	26	25
Weight	43.63	42.22	41.37	41.15	36.82	34.5	32.91	32.68	32.35	30.68

**Table 6:** Recognition accuracy of each channel subset based on KNN classifier (Unit: %).

Number of channels	1	2	3	4	5	6	7	8	9	10
Theta_Std+FE	85.93	93.58	96.03	96.72	97.07	99.45	99.27	99.33	99.27	99.42
Number of channels	11	12	13	14	15	16	17	18	19	20
Theta_Std+FE	99.27	99.40	99.30	99.33	99.38	99.33	99.28	99.38	99.35	99.32
Number of channels	21	22	23	24	25	26	27	28	29	30
Theta_Std+FE	99.37	99.30	99.30	99.20	99.32	99.23	99.32	99.32	99.30	99.23

**Table 7:** Comparison of optimal results.

Feature	Number of channels	Accuracy
Theta_Std	15	99.42%
FE	7	99.22%
Theta_Std+FE	6	99.45%

**Table 8:** Comparison of experimental results.

Methods	Number of channels	Accuracy
Theta_Std+FE+ReliefF_SFS (this paper)	6	99.45%
SE_KPCA [2]	30	98.33%
FE_FBN [25]	30	99.40%
SE_T_KPCA [26]	30	99.27%
CSPT_FBN [27]	7	99.17%
Adaptive multiscale FE [28]	2 (FP1, FP2)	95.37%
Multiscale FE based on the EMD [29]	2 (FP1, FP2)	87.50%

## Data Availability

The data that support the findings of this study is restricted as subjects' privacy.
